The article "The role of TMPRSS6/matriptase-2 in iron regulation and anemia" was published in 2014. Journal: Front Pharmacol.

# The role of *TMPRSS6*/matriptase-2 in iron regulation and anemia

**DOI:** 10.3389/fphar.2014.00114

**Published:** 2014-05-19

**Authors:** Chia-Yu Wang, Delphine Meynard, Herbert Y. Lin

**Affiliations:** ^1^Program in Anemia Signaling Research, Division of Nephrology, Program in Membrane Biology, Center for Systems Biology, Massachusetts General Hospital, Harvard Medical SchoolBoston, MA, USA; ^2^INSERM, U1043, CNRS, U5282, Université Paul Sabatier, Centre de Physiopathologie de Toulouse PurpanToulouse, France

**Keywords:** iron, *TMPRSS6*, matriptase-2, iron overload, IRIDA

## Abstract

Matriptase-2, encoded by the *TMPRSS6* gene, is a member of the type II transmembrane serine protease family. Matriptase-2 has structural and enzymatic similarities to matriptase-1, which has been implicated in cancer progression. Matriptase-2 was later established to be essential in iron homeostasis based on the phenotypes of iron-refractory iron deficiency anemia identified in mouse models as well as in human patients with *TMPRSS6* mutations. *TMPRSS6* is expressed mainly in the liver and negatively regulates the production of hepcidin, the systemic iron regulatory hormone. This review focuses on the current understanding of matriptase-2 biochemistry, and its role in iron metabolism and cancer progression. In light of recent investigations, the function of matriptase-2 in hepcidin regulation, how it is being regulated, as well as the therapeutic potential of matriptase-2 are also discussed.

## BIOCHEMISTRY OF MATRIPTASE-2

Type II transmembrane serine protease matriptase-2, encoded by the *TMPRSS6* gene, belongs to the family of type II transmembrane serine proteases (TTSP). Matriptase-2 is comprised of a transmembrane domain, followed by a sea urchin sperm protein, enteropeptidase and agrin (SEA) domain, a stem region containing two complement factor C1r/C1s, urchin embryonic growth factor and bone morphogenetic protein (CUB) domains and three low-density lipoprotein receptor (LDLR) class A repeats, and a C-terminal trypsin-like serine protease domain (Velasco et al., 2002; Ramsay et al., 2008). Matriptase-2 is synthesized as a single chain inactive proenzyme, which auto-activates itself by a cleavage at an arginine residue at the RIVGG consensus site between the prodomain and the catalytic domain (Ramsay et al., 2009b; Altamura et al., 2010). After the auto-activation, it remains membrane-bound through a single disulphide bond linking the pro- and catalytic domains (Ramsay et al., 2009a). Once the catalytic domain is released, it migrates as a single or dimeric species (Silvestri et al., 2008). Matriptase-2 shares high structural and enzymatic similarities with matriptase-1, which contains four LDLR repeats instead of three (Sanders et al., 2010), is expressed in epithelial cells, and has been implicated in the progression of cancers, such as breast, prostate, and colorectal cancer (Oberst et al., 2001; Velasco et al., 2002; Kang et al., 2003; Riddick et al., 2005).

The article "The role of TMPRSS6/matriptase-2 in iron regulation and anemia" was published in 2014. Journal: Front Pharmacol.

The structural features of matriptase-2 are highly conserved across mammalian species, including human, macaque monkey, dog, cow, mouse and rat, with human protein sharing >80% identity to matriptase-2 from other species (Ramsay et al., 2008). The expression pattern of *TMPRSS6* determined from mRNA expression studies and analysis of GenBank Unigene database indicates that matriptase-2 is predominantly expressed in the liver (Velasco et al., 2002; Finberg et al., 2008) but also to a lower extent in the kidney, spleen, brain, lung, mammary gland, testis, and uterus (Ramsay et al., 2008). In addition, aberrant expression of *TMPRSS6* is observed in different human cancers such as breast and prostate cancer (Parr et al., 2007; Sanders et al., 2008).

Matriptase-1, a close relative of matriptase-2, is known to be associated with two endogenous inhibitors: hepatocyte growth factor activator inhibitor (HAI)-1 and HAI-2, which inhibit matriptase-1 dependent activation of its physiological substrates, likely through an interaction with the second CUB domain (Szabo et al., 2008; Inouye et al., 2010). With 35% identity and structural similarities with matriptase-1 (Velasco et al., 2002), it is possible that matriptase-2 is also associated with an endogenous inhibitor. Indeed, Maurer et al. (2013) recently demonstrated that HAI-2 is a cognate inhibitor of matriptase-2 that inhibits its proteolytic activity, and thus increases hepcidin expression *in vitro*. However, the physiological role of HAI-2 in the regulation of hepcidin and iron metabolism remains to be investigated.

Following the identification and characterization of matriptase-2, Velasco et al. (2002) also examined the enzymatic activity of the catalytic serine protease domain against extracellular matrix components. It was found that matriptase-2 has the capacity to degrade fibronectin, fibrinogen, and type I collagen. Recently, membrane bound hemojuvelin has also been identified as a substrate for matriptase-2 *in vitro* (Silvestri et al., 2008), providing a straightforward mechanism for the effects of *TMPRSS6* mutations on hepcidin and iron regulations. However, as will be discussed below, evidence exists *in vivo* that is not consistent with this hypothesis.

## ROLE OF MATRIPTASE-2 IN IRON METABOLISM

Matriptase-2 is produced mainly by the liver and negatively regulates the production of hepcidin, the systemic iron regulatory hormone encoded by the *HAMP* gene (Du et al., 2008; Finberg et al., 2008). Hepcidin is a peptide secreted by the liver that plays a central role in adjusting iron absorption to meet iron needs of the body (Nicolas et al., 2001). Hepcidin negatively regulates cellular iron export by promoting the degradation of ferroportin (Nemeth et al., 2004), the only known iron exporter present on the surface of duodenal enterocytes, macrophages, and hepatocytes and thus limits iron absorption and iron release. It is now well established that *Hamp* expression is regulated by the bone morphogenetic protein (BMP)/sons of mothers against decapentaplegic (SMAD) signaling pathway (Babitt et al., 2006, 2007).

The article "The role of TMPRSS6/matriptase-2 in iron regulation and anemia" was published in 2014. Journal: Front Pharmacol.

At the molecular level, BMP6, the endogenous ligand of BMP/SMAD signaling, activates BMP-receptor complex by binding to type I and type II BMP receptors that induces phosphorylation (Andriopoulos et al., 2009; Meynard et al., 2009). The activated complex, in turn, phosphorylates Smad1,5,8/Smad4 complex, which then translocates to nucleus to modulate gene transcription (Wang et al., 2005; Babitt et al., 2006; Kautz et al., 2008). Hemojuvelin (HJV) acts as a coreceptor and is required to fully activate the BMP signaling ability (Babitt et al., 2006). The expression of BMP6 is proportional to hepatic iron concentrations and consistent with *Hamp* mRNA expression (Kautz et al., 2008).

## *TMPRSS6* MUTATIONS IN MICE AND HUMAN

Matriptase-2 regulates *Hamp* expression through the BMP/SMAD pathway (Finberg et al., 2010; Lenoir et al., 2011) in an as yet unfully characterized manner. Mice without functional matriptase-2 (both *mask* mice with truncated *Tmprss6* lacking the protease domain and *Tmprss6* knockout mice) showed a hypochromic microcytic anemia and an alopecia (Du et al., 2008; Folgueras et al., 2008). These phenotypes resulted from inappropriately high levels of *Hamp* mRNA expression (Du et al., 2008; Folgueras et al., 2008; Finberg et al., 2010).

Mutations in *TMPRSS6* in humans led to iron-refractory iron deficiency anemia (IRIDA) that is unresponsive to oral iron treatment and only partially responsive to parental iron therapy (Finberg et al., 2008). IRIDA is also characterized by congenital hypochromic, microcytic anemia, low mean corpuscular erythrocyte volume, low transferrin saturation, and defects in iron absorption and utilization (Finberg et al., 2008; Guillem et al., 2008; Melis et al., 2008). Currently, there are 42 different *TMPRSS6* mutations reported in humans, scattered throughout all the different extracellular domains (**Figure 1**).

**FIGURE 1:** ***TMPRSS6* gene structure and schematic representation of corresponding matriptase-2 mutations reported in IRIDA patients.** The genomic organization and the corresponding structural domains of matriptase-2 with currently identified mutations are shown. The missense, nonsense, frameshift and splice junction mutations are shown in green, blue, red and purple arrows, respectively. One in-frame deletion is boxed in gray. The mutations highlighted in red represent those appear to have haploinsufficiency.

The article "The role of TMPRSS6/matriptase-2 in iron regulation and anemia" was published in 2014. Journal: Front Pharmacol.

Interestingly, in contrast to current understanding of autosomal recessive disorder, haploinsufficiency is observed in some *TMPRSS6* mutations (**Figure 1**; Finberg et al., 2008; Pellegrino et al., 2012; Jaspers et al., 2013). Haploinsufficiency is also observed in animal models. Nai et al. (2010) reported that *Tmprss6* heterozygous knockout mice are more susceptible to iron deficiency compared to their wild-type littermates. Finberg et al. (2011) also demonstrated that, compared to mice deficient for *Hfe* alone, heterozygous loss of *Tmprss6* in *Hfe* knockout mice had higher hepcidin levels at 4 weeks of age, which presumably resulted in decreased hepatic iron concentrations at 8 weeks of age.

Human genome wide association studies (GWAS) highlighted the significance of matriptase-2 in control of iron homeostasis by identifying common *TMPRSS6* variants associated with abnormal hematological parameters, including hemoglobin, transferrin saturation, erythrocyte mean cell volume (MCV) and serum iron concentrations (Benyamin et al., 2009; Chambers et al., 2009; Tanaka et al., 2010). Following GWAS, population-based cohort studies were investigated in China and Italy to study the association between serum iron parameters, iron-related diseases and specific *TMPRSS6* single nucleotide polymorphisms (SNPs): rs855791 (V736A) and rs4820268 (D521D). It was found that *TMPRSS6* SNPs was associated with lowered serum iron, hemoglobin, and plasma ferritin levels, consistent with lowered risk of iron overload and increased risk of iron deficiency anemia in Chinese population (An et al., 2012; Gan et al., 2012). A retrospective cohort study in northern Italy also suggested that *TMPRSS6* V736A polymorphism is likely to be a gene modifier in hemochromatosis patients, influencing the susceptibility of cirrhosis (Valenti et al., 2012). Nai et al. (2011) demonstrated that *TMPRSS6* V736A directly modulates *HAMP* expression *in vitro* and that healthy individuals with the homozygous substitution had lower levels of serum hepcidin, higher serum iron and higher transferrin saturation. Taken together, these studies clearly establish *TMPRSS6*/matriptase-2 as an important regulator of iron homeostasis in humans. A recent review focused more on the anemia induced by matriptase-2 mutations is complementary to the current review (De Falco et al., 2013).

The article "The role of TMPRSS6/matriptase-2 in iron regulation and anemia" was published in 2014. Journal: Front Pharmacol.

## FUNCTION OF MATRIPTASE-2 IN HEPCIDIN REGULATION

Matriptase-2 inhibition of hepcidin activation by cleaving membrane hemojuvelin has been established *in vitro* (Silvestri et al., 2008). When overexpressed in HeLa cells, matriptase-2 interacts and induces the cleavage of membrane hemojuvelin at the cell surface, resulting in the generation of soluble hemojuvelin that is released into the cell medium (Silvestri et al., 2008). However, in both *mask* and *Tmprss6* knockout mice, hepatic hemojuvelin levels at the membrane were found unexpectedly to be decreased, compared to wild-type animals (Krijt et al., 2011; Frydlova et al., 2013). In addition, the levels of serum soluble hemojuvelin, which one would expect to be decreased in *Tmprss6* knockout, did not differ from wild-type mice (Chen et al., 2013). Although the possibility that soluble hemojuvelin and fragments are rapidly degraded *in vivo* cannot be excluded, these data suggested that hemojuvelin may not be the endogenous substrate of matriptase-2 and that matriptase-2 functions in a more complicated way *in vivo* than by merely cleaving hemojuvelin to regulate hepcidin and iron.

Several studies have been conducted to study the role of matriptase-2, by crossing *Tmprss6* knockout mice with several iron overload mouse models, including the generations of *Hjv/Tmprss6*, *Bmp6/Tmprss6*, *Hfe/Tmprss6*, and *Tfr2/Tmprss6* double mutant mice (Truksa et al., 2009; Finberg et al., 2011; Lenoir et al., 2011; Lee et al., 2012). In mice lacking both *Hjv* and *Tmprss6*, *Id1*, a target gene of BMP6 signaling, and *Hamp* mRNA levels were low, whereas serum iron, transferrin saturation, and liver iron concentration were high, similar to phenotypes of mice deficient for *Hjv* alone (Truksa et al., 2009; Finberg et al., 2010). These results indicate that if the substrate of matriptase-2 is downstream of hemojuvelin, it is likely to be along the SMAD signaling pathway. It is known that inflammatory cytokines, such as LPS and IL6, can induce *Hamp* expression in the absence of *Hjv* (Niederkofler et al., 2005), presumably via the Stat3 and Stat5 pathways (Verga Falzacappa et al., 2007; Meynard et al., 2013). However, it was surprising to find that the lack of both *Hjv* and *Tmprss6* in mice did not impair the responsiveness of hepcidin to BMP2 and IL6, but did fail to respond to iron challenge (Truksa et al., 2009). In mice deficient for both *Bmp6* and *Tmprss6*, the levels of *Hamp* and *Id1* mRNAs did not differ from mice deficient for *Bmp6* alone; however, their plasma iron levels and hepatic iron stores were significantly lower, suggesting the loss of matriptase-2 ameliorates iron overload conditions in *Bmp6* knockout mice (Lenoir et al., 2011). It is unclear why *Bmp6/Tmprss6* mice had less iron loading compared to mice deficient for *Bmp6* alone, but *Hamp* mRNA levels did not differ between *Bmp6/Tmprss6* and *Bmp6* knockout mice. Whether matriptase-2 has a significant role besides effects on BMP/SMAD signaling in iron metabolism, remain to be investigated.

The article "The role of TMPRSS6/matriptase-2 in iron regulation and anemia" was published in 2014. Journal: Front Pharmacol.

Mice deficient for *Hfe* or *Tfr2* alone also develop iron overload phenotypes with inappropriately low *Hamp* mRNA expression and high serum iron parameters, compared to wild-type animals (Ahmad et al., 2002; Wallace et al., 2005). It is suggested that *Hfe* competes with transferrin for binding to transferrin receptor-1 and thus inhibits *Hamp* expression (Giannetti and Bjorkman, 2004; Schmidt et al., 2008). Others also showed that *Hfe* knockout mice had high *Bmp6* mRNA expression but inappropriately low Smad1/5/8 phosphorylation, suggesting *Hfe* facilitates signal transduction initiated by BMP6 (Corradini et al., 2009; Kautz et al., 2009). However, the underlying mechanisms of how *Hfe* and Tfr2 contribute in BMP/SMAD signaling pathway is unclear. Mice deficient for both *Hfe* or *Tfr2* and *Tmprss6*, had high *Hamp* mRNA expression and exhibited iron deficiency microcytic anemia mimicking the phenotypes of mice lacking functional matriptase-2 alone (Finberg et al., 2011; Lee et al., 2012). This suggests that *Hfe* and Tfr2, if involved in BMP/SMAD pathway, are likely to be upstream of matriptase-2 signaling.

## REGULATION OF MATRIPTASE-2

Studies have shown that matriptase-2 expression can be modulated by iron status (Meynard et al., 2011; Zhang et al., 2011). In rats under acute iron deprivation, hepatic matriptase-2 protein levels are upregulated to repress hepcidin production (Zhang et al., 2011). Interestingly, matriptase-2 levels are also increased in response to chronic iron treatment and BMP6 administration in mice, possibly to prevent excessive hepcidin production, suggesting a dual role of matriptase-2 in the maintenance of tight systemic iron balance in response to iron (Meynard et al., 2011). In addition, studies also suggest that *TMPRSS6* mRNA expression is suppressed by conditions of inflammation (Meynard et al., 2013) and is upregulated in hypoxia (Lakhal et al., 2011; Maurer et al., 2012) and by erythropoietin (Peng et al., 2010). Human hepatoma Hep3B cells treated with interleukin-6 and mice injected with lipopolysaccharide demonstrated a downregulation of *TMPRSS6* via a decrease in Stat5 phosphorylation, independent of BMP/SMAD pathway (Meynard et al., 2013). Studies using Hep3B cells revealed that *TMPRSS6* is upregulated by HIF-1α and HIF-2α. This upregulation resulted in a decrease in membrane hemojuvelin and thus reducing hepcidin production (Lakhal et al., 2011). In mice, *Tmprss6* mRNA expression is induced by erythropoietin (Peng et al., 2010), which is also shown to be a negative regulator of hepcidin expression (Sasaki et al., 2012). Whether the downregulation of hepcidin by erythropoietin is dependent on *Tmprss6* or through other unidentified mechanisms remains to be investigated.

The article "The role of TMPRSS6/matriptase-2 in iron regulation and anemia" was published in 2014. Journal: Front Pharmacol.

## MATRIPTASE-2 AS A THERAPEUTIC TARGET

Genetic studies of mice deficient for both *Tmprss6* and *Hfe* or *Tfr2* or *Hbb*^th3/^^+^, the mouse model of β-thalassemia intermedia, have shown that iron overload can be prevented by targeting *Tmprss6* (Finberg et al., 2011; Lee et al., 2012; Nai et al., 2012). It is believed that the therapeutic effect did not come from silencing *Tmprss6* directly but from increased hepcidin production, resulting in lowered circulating iron burden (Camaschella, 2013). Studies targeting *Tmprss6* in *Hbb^th3/+^* and *Hfe* knockout mice by injecting silencing RNA (Schmidt et al., 2013) and anti-sense oligonucleotides (Guo et al., 2013) have successfully suppressed *Tmprss6* mRNA expression, leading to elevated hepcidin levels, improved iron overload in *Hfe* knockout and anemia and β-thalassemic mice. It is unclear how the ineffective erythropoiesis is improved by dampening *Tmprss6* expression in *Hbb^th3/+^* mice. However, higher hepcidin level inhibiting iron delivery to the erythroid precursors seems to play a role as evident by the similar effects achieved by overexpression of *Hamp*, iron restriction, and the injection of transferrin to *Hbb^th3/+^* mice (Gardenghi et al., 2010; Li et al., 2010; Finberg, 2013).

One limitation of using this method is that, unlike traditional phlebotomy and chelation therapies, iron is not removed or excreted from the body, and therefore, may not be an ideal treatment for patients with severe iron overload and transfusion-dependent thalassemia (Camaschella, 2013). It could, however, improve therapeutic efficacy when used in combination with other traditional therapies by preventing intestinal iron absorption. A key issue for the use of RNA interference for clinical applications is the delivery method. There are safety concerns with viral vectors and non-viral delivery methods, which are still in their early development stage. Concerns have also been raised regarding the potential for off-target effects of siRNAs and their possible induction of interferon-stimulated genes. Other novel inhibitors of *TMPRSS6*, such as small molecule inhibitors, once identified, may eventually become useful therapeutic agents as well.

The article "The role of TMPRSS6/matriptase-2 in iron regulation and anemia" was published in 2014. Journal: Front Pharmacol.

## ROLE OF MATRIPTASE-2 IN CANCER

Numerous members of the type II transmembrane serine protease family have been associated with a variety of different human cancers due to the differential expression patterns observed in these proteases between normal and cancerous tissues and cells (Webb et al., 2011). However, there are only a limited number of studies examining the involvement of matriptase-2 in human cancer, including breast cancer (Hartikainen et al., 2006; Parr et al., 2007; Tuhkanen et al., 2013) and prostate cancer (Sanders et al., 2008; Webb et al., 2012).

The association between matriptase-2 and breast cancer was established by a case control study in eastern Finnish population where they found a SNP (rs733655) in *TMPRSS6* gene associated with increased breast cancer risk (Hartikainen et al., 2006). It was later shown that *TMPRSS6* mRNA expression inhibits breast tumor development and thus correlates with favorable prognostic outcome in patients (Parr et al., 2007). Recently, Tuhkanen et al. (2013) also demonstrated the association of several *TMPRSS6* variants with breast cancer risk and survival. It was highlighted that matriptase-2 protein levels decrease with tumor progression, and lower gene expression is seen in poor-prognosis-related triple-negative breast cancers (Tuhkanen et al., 2013). Mastriptase-2 is also implicated in tumor invasion and metastasis in prostate cancer *in vitro* (Sanders et al., 2008; Webb et al., 2012). These results indicate the involvement of matriptase-2 in tumor development. However, it is not clear whether the role of *TMPRSS6* in cancer progression is due to its ability to cleave extracellular matrix component such as fibronectin or due to a modification of iron parameters in cancer cells.

*TMPRSS6* expression is predominantly found in low invasive breast cancer cell lines such as MCF-7 and is absent in more invasive breast cancer cell lines such as MDA-MB-231 (Parr et al., 2007). Overexpression of matriptase-2 in MDA-MB-231 leads to a reduction of invasiveness and motility of the transfected cells and suppresses their tumorigenesis when xenografted in athymic nude mice suggesting that matriptase-2 could be involved in cancer progression through its capacity to cleave extracellular matrix components (Parr et al., 2007). However, variations of the iron status and iron regulatory genes expression were not addressed in the transfected cells in this study.

Many cancers exhibit an increased requirement for iron, presumably because of the need for iron as a cofactor in proteins essential to sustain growth and proliferation. The iron exporter ferroportin is expressed in breast cancer cells. Pinnix et al. (2010) showed that cells with high hepcidin and low ferroportin levels tended to be more aggressive. They concluded that having a breast cancer with low hepcidin and high ferroportin levels is an independent predictor of prognosis for a >90% 10-year survival rate (Pinnix et al., 2010), however, the mechanism is still to be investigated. Further studies are required to clarify the role of matriptase-2 in cancer progression.

The article "The role of TMPRSS6/matriptase-2 in iron regulation and anemia" was published in 2014. Journal: Front Pharmacol.

## Conflict of Interest Statement

The authors declare that the research was conducted in the absence of any commercial or financial relationships that could be construed as a potential conflict of interest.
